# Network Pharmacology Analysis, Molecular Docking, and *In Vitro* Verification Reveal the Action Mechanism of *Prunella vulgaris* L. in Treating Breast Cancer

**DOI:** 10.1155/2022/5481563

**Published:** 2022-08-10

**Authors:** Haotian Bai, Rui Wang, Yalan Li, Xiao Liang, Junhao Zhang, Na Sun, Jing Yang

**Affiliations:** ^1^College of Pharmacy, Heilongjiang University of Chinese Medicine, Harbin, Heilongjiang 150040, China; ^2^Key Laboratory of Basic and Application Research of Beiyao, Heilongjiang University of Chinese Medicine, Ministry of Education, Harbin, Heilongjiang 150040, China; ^3^College of Basic Medical Science, Heilongjiang University of Chinese Medicine, Harbin, Heilongjiang 150040, China

## Abstract

**Background:**

*Prunella vulgaris* L. is effective in the treatment of breast cancer (BRCA); however, the underlying mechanism is still unclear. The aim of this study was to elucidate the mechanism of treatment of BRCA by *P. vulgaris* using network pharmacology and molecular docking technology, and to verify the experimental results using human BRCA MDA-MB-231 cells.

**Methods:**

Active components and action targets of *P. vulgaris* were determined using the TCMSP™, SwissTarget Prediction™, and TargetNet™ databases. GeneCards™ and OMIM™ provided BRCA targets. After obtaining common targets, a protein-protein interaction (PPI) network was constructed using the STRING™ database, and Gene Ontology and Kyoto Encyclopedia of Genes and Genomes (KEGG) pathway analyses were conducted using the Xiantao™ academic database. Cytoscape™ was used to construct “single drug-disease-component-target” and “single drug-disease-component-target-pathway” networks. The Human Protein Atlas™ was used to determine protein expression levels in BRCA cell lines. AutoDock tools™ were used to carry out molecular docking for the first 10 targets of quercetin and the PPI network. Finally, the abovementioned results were verified using cell experiments.

**Results:**

We obtained 11 active components, 198 targets, and 179 common targets, including DUOX2, MET, TOP2A, and ERBB3. The results of KEGG pathway analysis screened 188 related signaling pathways and indicated the potential key role of PI3K-Akt and MAPK signaling pathways in the antibreast cancer process of *P. vulgaris*. The results of molecular docking showed that the first 10 targets of quercetin interacted well with the protein network. Cell experiments showed that quercetin effectively inhibited the proliferation of MDA-MB-231 cells by regulating apoptosis and cell cycle, which may be partly related to the MAPK signaling pathway.

**Conclusion:**

Synergistic effects of multiple components, targets, and pathways on the anti-BRCA activity of *P. vulgaris* could provide a theoretical basis for further study on its complex anti-BRCA mechanism.

## 1. Introduction

In recent years, the incidence rate of breast cancer (BRCA) has been increasing worldwide, at a rate of 3% per year [1]. Therefore, BRCA is becoming the cancer with the fastest growing incidence rate among women [2]. Simultaneously, the age of onset of BRCA is also gradually decreasing, causing a great psychological burden on the patients, making patients and their families bear great economic and life pressure, and seriously reducing people's happiness levels [3]. According to the International Cancer Institute of WHO, the incidence rate of BRCA worldwide was 24.2% and the mortality rate was 15.0% by 2018 [4]. At present, the treatment of BRCA mainly involves a combination of surgery, chemotherapy, and radiotherapy. However, the abovementioned methods present several limitations. The treatment of breast disease affects the health of other systems and leads to complications such as slow wound recovery, changes in body shape, liver and kidney injury, changes in metabolism, and severe alopecia. BRCA adversely affects women physically and mentally [5, 6]. Therefore, treatments with few adverse reactions and wide applications need to be developed. Traditional Chinese medicine treatment presents great potential owing to its characteristics of small adverse reactions and a good curative effect. The occurrence, development, invasion, and metastasis of BRCA is a complex process. Traditional Chinese medicine is an important way to treat BRCA, regardless of the stage.

The dried ear of *Prunella vulgaris* L, a perennial herb in the family Lamiaceae, has a medicinal and edible homology. It has a medicinal history of thousands of years and was first mentioned in the Shennong herbal classic. Its Chinese name means “grass will wither after the summer solstice.” *Prunella vulgaris* is bitter, spicy, and cold, and it acts along the liver and gallbladder meridians. It can clear the liver and dissipate fire, clear eyesight, dissipate nodules, and disperse swelling [7], pain, photophobia, dizziness, vertigo, gall, BRCA, hypertension, lymphatic tuberculosis, infiltrative pulmonary tuberculosis, simple goiter, mumps, acute icteric infectious hepatitis, and other diseases with a good clinical therapeutic effect [8–11]. Modern research shows that the water, alcohol, and ethyl acetate extracts of *P. vulgaris* have various pharmacological effects, including antitumor, antibacterial, anti-inflammatory, immunosuppressive, free radical scavenging, antioxidative, and antiviral properties [12–14]. With the gradual deepening of research on *P. vulgaris* and its extract, its related pharmacological effects are being gradually clarified, and clinical research on it is becoming increasingly extensive.

Network pharmacology is a recently introduced analytical method. It conducts “multitarget and multipathway” analysis of drugs and diseases by integrating various databases and constructs a “drug active ingredient disease” model to visually analyze the studied action mechanism and comprehensively predict the targets [15]. Though *P. vulgaris* has been shown to be clinically effective in the treatment of BRCA in a vast number of studies, its underlying mechanism is unclear. This study aimed to predict the potential components, targets, and molecular pathways of *P. vulgaris* against BRCA based on network pharmacology. Furthermore, we used molecular docking and cell experiments to verify and provide a theoretical basis for the potential mechanism (Figure 1).

## 2. Materials and Methods

### 2.1. Collection of Active Components and Action Targets of *P. vulgaris*

The TCMSP database and analysis platform (https://tcmspw.com/tcmsp.php) were used to get self-healing active ingredients and potential targets [16]. Taking “*Prunella vulgaris* L” as the retrieval word, oral bioavailability (OB) ≥ 30% and drug-likeness (DL) ≥ 0.18 are assumed as the screening conditions, and the eligible active ingredients are collected [17]. The corresponding targets were obtained according to the screened active ingredients of *Prunella subtilis*. Using the UniProt database (https://www.uniprot.org/) [18], the species was defined as “*Homo sapiens*,” and the gene names corresponding to the targets of the active ingredients of *Prunella subtilis* were collected. From the PubChem database (https://pubchem.ncbi.nlm.nih.gov/) [19], in chemical structure of the linear canonical SMILES, import the component target database (SwissTargetPrediction, https://www.swisstargetprediction.ch/) [20], the choice of species for human *Homo sapiens*, and potential acquisition targets. Then, using the UniProt specification TargetNet of targets, the chemical composition of the canonical SMILES number was entered into TargetNet (https://targetnet.scbdd.com/), prob >0 genes were selected, and used the UniProt specification TargetNet of targets. The targets of the three databases were merged and the duplicate targets were deleted.

### 2.2. Collection of Potential Targets for BRCA

Using the GeneCards database (https://www.genecards.org/) (correlation score ≥1.0) [21] and the OMIM database (https://www.omim.org/) [22], using “BRCA” as a retrieval term, potential targets for BRCA were retrieved. After removing the duplicate genes, the targets associated with BRCA were eventually collected.

### 2.3. Construction of a “Single-Substance Drug-Disease-Component-Target” Network

The common targets of *P. vulgaris* and BRCA were obtained from the Xiantao academic database (https://www.xiantao.love), and the Wayne map was drawn using the Venny plate. The “single-substance drug-disease-component-target” network was constructed using Cytoscape 3.7.1 software.

### 2.4. Construction of the PPI Network

Using STRING database (https://string-db.org/), the PPI network was constructed. The target points of *P. vulgaris* and BRCA obtained in previous step were introduced into the STRING database, the species “*Homo sapiens*” was defined, and the confidence level was >0.4. The light blue line represents the interprotein interaction from the database and the purple line represents the protein intercropping verified by experiments. GraphPad prism 7.0 was used to display the adjacent number of the top 35 proteins in the PPI network.

### 2.5. Analysis of Pathways and Functional Enrichment

To further study the molecular mechanism of *P. vulgaris* against BRCA, GO and KEGG pathway analyses were carried out using the Xiantao academic database (https://www.xiantao.love). The top 10 biological processes, molecular functions, cellular components, and KEGG pathways were selected (*P* < 0.05), and the results were visualized by GraphPad prism 7.0. Then, the experimental data such as active ingredients, targets, and the top 10 KEGG pathways were imported into Cytoscape 3.7.1 software to construct a “single-substance drug-disease-component-target-pathway” network.

### 2.6. Molecular Docking Analysis

For further verification, quercetin, a key active component of *P. vulgaris*, was selected for molecular docking with the top 10 targets in the PPI network. The 2D structure of quercetin was downloaded using the PubChem database (https://www.ncbi.nlm.nih.gov/Pccompound/) and saved in an SDF format file. The SDF format file of quercetin was modified by ChemBio3D software to minimize its structural energy and save it in a mol format. From the PDB database (https://www.pdb.org/), the crystal structure of the target was downloaded and PyMOL software was used for pretreatment, including water molecule removal and hydrogenation. Then, the 3D structure and target crystal structure of quercetin were converted into PDBQT format files using Autodock Tools, and the molecular docking was carried out by AutoDock Vina software. The binding activity between quercetin and the target was evaluated by binding energy. Finally, PyMOL software was used to visualize the docking file.

### 2.7. Validation of the “Target Pathway”

To further verify the important role of the screened pathways and targets in *P. vulgaris* in the treatment of BRCA, the selected important pathways were input into the KEGG database (https://www.kegg.jp/). The role of the screened target in this pathway is queried and displayed in the human protein map database (https://www.proteinatlas.org/). The final verification of the screened target genes is carried out to verify whether they are enriched in BRCA tissues and cells, so as to provide a sufficient theoretical basis for future studies.

### 2.8. Experimental Verification

#### 2.8.1. Experimental Drugs and Cells

Human BRCA MDA-MB-231 cells were purchased from Shanghai Fu Heng Biotechnology Co., Ltd., and quercetin (purity >97%) was purchased from Shanghai McLean Biological Co., Ltd.

#### 2.8.2. Experimental Reagents and Instruments

  Fetal bovine serum© (GIBCO Co., Ltd)
  L15 Medium© (GIBCO Co., Ltd)
  3-(4,5-dimethylthiazol-2-yl)-2,5-diphenyltetrazolium bromide (MTT)© (Solarbio Co., Ltd)
  ERBB3 polyclonal antibody© (Bio-swarm Co., Ltd)
  MET polyclonal antibody© (Bio-swarm Co., Ltd)
  Cleaved poly ADP-ribose polymerase© (Cleaved PARP) (Abways Co., Ltd)
  Cleaved caspase-3© (Abways Co., Ltd)
  p38 polyclonal antibody© (Bio-swarm Co., Ltd)
  Glyceraldehyde-3-phosphate dehydrogenase (GAPDH) polyclonal antibody© (Bio-swarm Co., Ltd)
  Secondary antibody sheep antirabbit IgG© (Abways Co., Ltd)
  Bicinchoninic acid (BCA) protein detection kit© (Bio-swarm Co., Ltd)
  Emitter coupled logic (ECL) chemiluminescence kit© (SANGON biotech Co., Ltd)
  Pennexin V apoptosis detection kit I cell apoptosis kit© (Elabscience Co., Ltd)
  Cell cycle detection kit© (Elabscience Co., Ltd)
  ELX800 chemiluminescence enzyme labeling instrument® (Beijing Liuyi Co., Ltd)
  DYCZ-24DN double vertical electrophoresis instrument® (Beijing Liuyi Co., Ltd)
  DYCZ-40D transfer electrophoresis instrument® (Beijing Liuyi Co., Ltd)
  Clinxchemiscope 6000 chemiluminescence instrument® (Shanghai Qinxiang Co., Ltd.)
  Facscantoii flow cytometry® (BD Co., Ltd.)

#### 2.8.3. MTT Cell Proliferation Test

The effect of quercetin on the proliferation of human BRCA MDA-MB-231 cells was detected using the MTT method. Logarithmically grown MDA-MB-231 cells were inoculated into 96-well plates (5 × 10^4^ well^−1^), 5 multiple wells in each group. After 12 h of cell adhesion, 0, 10, 20, 30, 40, and 50 *μ*g/mL were added, respectively. Quercetin was treated for 24 or 48 h, respectively, and the cell morphology was observed. After treatment with quercetin for 24 or 48 h, a 5 mg/mL MTT solution was added to each well and incubated in the cell incubator for 4 h. Carefully suck and discard the culture supernatant in the well, add 150 *μ*L of dimethyl sulfoxide to each well, and oscillate at low speed in the dark at room temperature for 10 min to fully dissolve the crystal. The optical density (OD) of each well was measured by using a microplate reader at 570 nm. The relative cell viability and cell inhibition rate were calculated with reference to the OD of the blank control group.

#### 2.8.4. Flow Cytometry

The effect of quercetin on the cell cycle and apoptosis of human BRCA MDA-MB-231 cells was detected using flow cytometry. Logarithmically grown MDA-MB-231 cells were inoculated into 96-well plates (5 × 10^4^/well). MDA-MB-231 cells were treated with quercetin at different concentrations for 24 h, digested with trypsin, and collected. Cell cycle analysis was carried out. After the abovementioned treatment, the cells were centrifuged at 1500 rpm for 5 min. After that, 1 mL of phosphate buffered saline (PBS) was added for cleaning and centrifugation, and the supernatant was sucked out. Then, 2 mL of 75% ethanol was added and fixed overnight at 4°C. The supernatant was then centrifuged and removed, and the cells were resuspended twice with PBS. Finally, a 500 mL mixture of propidium iodide (PI) and ribonuclease (RNaseA) was prepared in each tube. After being kept away from light at 37°C for 30 min, the cell cycle was detected by flow cytometry. After the abovementioned treatment, the cell density was adjusted to 1 × 10^5^ L^−1^. Then, 100 *μ*L of binding buffer was added to each tube to resuspended the cells. Furthermore, 5 *μ*L of annexin v-phycoerythrin (annexin V-PE) and 5 *μ*L of 7-amino-actinomycin D (7-AAD) were added and mixed well. Then, it was incubated at room temperature in the dark for 20 min. Finally, the cells were washed with PBS, and 500 *μ*L of PBS was added to resuspend the cells to detect apoptosis by flow cytometry.

### 2.9. Western Blotting

After the abovementioned treatment, human BRCA MDA-MB-231 cells were added to the protein lysate and lysed for 30 min on ice. The total protein concentration was measured using the bicinchoninic acid (BCA) assay. Sodium dodecyl sulfate-polyacrylamide gel electrophoresis (SDS-PAGE) was used to separate 20 *μ*g of protein at 100 V on ice for 2 h, before transferring onto the polyvinylidene fluoride (PVDF) membrane. The PVDF membrane was transferred to skimmed milk powder containing 5%, and the membrane was shaken on a decolorization shaker for 1 h at room temperature. The membrane was removed from the blocking solution, placed in a hybridization bag, and the following specific primary antibodies were added: cleaved caspase-3 (1 : 1000), or cleaved PARP (1 : 1000), or ERBB3 (1 : 1000), or MET (1 : 1000), or p38 (1 : 1000), and GAPDH (1 : 5000). After incubation at 4°C overnight, wash with Tris buffered saline tween (TBST) on a decolorizing shaker at room temperature 3 times for 8 minutes each time. The membrane was incubated in secondary antigoat antirabbit IgG (1 : 2000) at room temperature for 1 h and washed on a decolorizing shaking table with TBST 3 times at room temperature for 8 min each time. ECL chemiluminescence developing drops were added onto the PVDF film, the film was put into a chemical imaging analyzer for exposure, and photos were taken. ImageJ 1.4.1 software was used to collect the gray value of the protein and to conduct semiquantitative analysis.

## 3. Results

### 3.1. Collection of Active Components and Action Targets of *P. vulgaris*

A total of 242 active components of *P. vulgaris* were obtained in the Traditional Chinese Medicine Systems Pharmacology (TCMSP) database. Based on the screening criteria of OB ≥ 30% and DL ≥ 0.18, 11 potential active components were obtained, all of which were terpenoids and sterols. To facilitate the follow-up study, these components were numbered PL1–PL11 (Table 1). Subsequently, 791 potential targets related to *P. vulgaris* were obtained from the TCMSP database. The UniProt database was used to correct the target gene name and remove invalid and duplicate values. Finally, 198 targets were obtained.

### 3.2. Collection of Potential Targets for BRCA

Using the GeneCards and OMMI databases, 150 and 21510 BRCA targets were obtained, respectively. Combined with the elimination of duplicate values, 15231 BRCA potential targets were obtained.

### 3.3. Construction of the “Single-Substance Drug-Disease-Ingredient-Target” Network

The 198 target sites of *P. vulgaris* collected were matched with 15231 potential targets of BRCA. Using the Xiantao academic database, 179 common targets of *P. vulgaris* and BRCA were identified, and a Venn map was plotted using the Wayne chart (Figure 2). Only eight effective components of *P. vulgaris* corresponding to the selected common target were found, and three effective components (PL7–9; cactus flavin-i, monoglucoside, and stigmasterol) were excluded. The active ingredients of *P. vulgaris* and the common target of *P. vulgaris* and BRCA were introduced into Cytoscape 3.7.1 software to build the single-substance drug-disease ingredient-target network (Figure 3). The network has 188 nodes, including *P. vulgaris* (light red round), 8 active ingredients screened from *P. vulgaris* (purple triangle), and 179 *P. vulgaris* and common target nodes of BRCA (light green and green ellipse). Quercetin is the most active component of *P. vulgaris* against BRCA. It is directly related to 59 targets, such as DUOX2, MET, TOP2A, ERBB3, and the interleukin family (IL-2, IL-4, IL-6, IL-1A).

### 3.4. Construction of Protein-Protein Interaction Network (PPI)

Twenty-five common targets of *P. vulgaris* and BRCA were introduced into the STRING database, and the species “*Homo sapiens*” was defined and screened with a confidence level >0.4. The resulting PPI network had 175 nodes, representing all prediction targets (Figure 4). The edge line represents the relationship between the targets, and the important relationship of the represented proteins in this network can be intuitively judged by the size of the circular area. Among them, the interacting proteins with a comprehensive numerical score >0.95 include MET-DUOX2, TOP2A-ERBB3, DUOX2-TOP2A, and SCN5A-MAP2. The interaction between these proteins plays an important role in the network. GraphPad prism was used to visualize the number of top 35 adjacent targets in the network and to draw a histogram (Figure 5). The results show that SCN5A, MAP2, DUOX2, and TOP2A are the core targets, and the number of adjacent targets is 2016, 1827, 1548, and 1531, respectively.

### 3.5. Pathway Enrichment Analysis

In order to further study the mechanism of *P. vulgaris* against BRCA, Gene Ontology (GO) and Kyoto Encyclopedia of Genes and Genomes (KEGG) pathway analysis of 179 common targets of *P. vulgaris* and BRCA were carried out using the Xiantao academic database. A total of 2905 GO enrichment entries was obtained, including 2573 biological process entries, 224 molecular functions, and 108 cellular components. In the biological process, *P. vulgaris* was mainly involved in (GO: 0007188 *n* = 42), lipopolysaccharide (GO: 0032496, *n* = 40), reaction to the bacterial source (GO: 0002237, *n* = 40), reaction to the metal ions (GO: 0010038, *n* = 39), and cell response to drugs (GO: 0035690, *n* = 39). *P. vulgaris* was mainly related to membrane raft (GO: 0045121, *n* = 30), membrane microdomain (GO: 0098857, *n* = 30), membrane region (GO: 0098589, *n* = 30), transcription factor complex (GO:0005667, *n* = 17), and plasma membrane raft (GO: 0044853, *n* = 15). In the process of molecular function enrichment, *P. vulgaris* was linked with ubiquitin-like protein ligase (GO: 0044389, *n* = 19), endopeptidase activity (GO: 0004175, *n* = 18), DNA binding transcriptional activator activity and RNA polymerase II specificity (GO: 0001228, *n* = 18), receptor ligand activity (GO: 0048018, *n* = 18), and cytokine receptor binding (GO: 0005126, *n* = 17), which have a great impact. According to *P* < 0.05, the top 10 GO enrichment entries were screened and visualized by GraphPad prism (Figure 6). Using the KEGG pathway analysis, the common constituents were gathered into 188 signaling pathways. *P. vulgaris* was mainly involved in the PI3K-Akt signaling pathway (hsa04151, *n* = 30), MAPK signaling pathway (hsa04010, *n* = 29), hepatitis B (hsa05161, *n* = 32), human cytomegalovirus infection (hsa05163, *n* = 31), and the signaling pathway of the diabetes in the complication of diabetes mellitus. According to *P* < 0.05, the top 10 pathways were screened out and visualized by GraphPad Prism (Figure 7). Finally, the results of the effective ingredients of *P. vulgaris*, the common target of *P. vulgaris* and BRCA, and the top 10 KEGG signaling pathways were imported into Cytoscape software to construct a “single-substance drug-disease-ingredient-target pathway” network (Figure 8). The network has 199 nodes, including *P. vulgaris* (pale blue hexagon), BRCA (light purple octagon), 8 active ingredients of *P. vulgaris* (light pink hexagon), 179 *P. vulgaris* and BRCA common targets (light yellow diamond), and the top 10 signal pathways (light green V font). From this picture we can see quercetin (PL11). Multipurpose targets are the core components of *P. vulgaris* against BRCA. This network map directly reflects the mechanism of *P. vulgaris* against BRCA through multicomponent, multitarget, and multichannel.

### 3.6. Molecular Docking Analysis

Combining the “component core” target network with the PPI network, the gene targets were sorted at the degree level, and the first ten key targets (ERBB3, INSR, MET, NCOA1, NCOA2, COL3A1, TOP2A, DUOX2, MAP2, and SCN5A) were selected for molecular docking with *P. vulgaris* for the treatment of BRCA. Using AutoDock Vina software, quercetin was docked with the top 10 targets in the PPI network, and the binding activity of components and targets was evaluated by the binding energy. It is generally believed that binding energy < −4.52 kcal/mol indicates that there is a certain binding activity between ligand small molecules and receptor proteins; binding energy < −5.0 kcal/mol showed that they had a good binding activity; binding energy < −7.0 kcal/mol indicates that the ligand has a strong binding activity with the receptor [23]. Molecular docking results showed that all binding energies were greater than 4.52 kcal·mol^−1^, indicating that quercetin was well docked with these targets (Table 2). PyMOL software was used to visually analyze the molecular docking results of quercetin with DUOX2 (PDB ID: AF), ERBB3 (PDB ID: 3kex), TOP2A (PDB ID: 4r1f), and MET (PDB ID: 2rfs) (Figure 9). As shown in Figure 9, quercetin interacts with amino acid residue ARG-241 of TOP2A through a hydrogen bond. Two hydrogen bonds were observed between quercetin and the amino acid residue PHE-1490 of DUOX2. Quercetin forms hydrogen bonds with ARG-1208 and ASN-1209 on the key residues of the active site. Quercetin interacts with amino acid residues ASP-833 and THR-768 of ERBB3 through hydrogen bonds.

### 3.7. Target Pathway Validation Analysis

Previous KEGG pathway analysis revealed that the PI3K-Akt and MAPK pathways were crucial in the process of *P. vulgaris* in the treatment of BRCA. Therefore, the abovementioned two pathways were further validated. The names of the two pathways were entered into the KEGG database, and the target selection points (DUOX2, ERBB3, MET, and TOP2A) were entered into the target plate. The results of further analysis are shown in Figure 10. ERBB3 and MET proteins are enriched in the cell membrane and act through the classical MAPK pathway. It is shown by cBioPortal database analysis (Figure 11). ERBB3 and MET were found to be highly expressed in BRCA. Therefore, through the final verification, the important mechanism of anti-BRCA is clear.

### 3.8. Quercetin Inhibits Proliferation of Human BRCA MDA-MB-231 Cells

The effect of quercetin with different concentrations on the proliferation of the human BRCA cell line MDA-MB-231 was detected using the MTT method at 24 or 48 h (Figure 12(a)). Quercetin significantly inhibited the proliferation of human BRCA MDA-MB-231 cells in a time and dose-dependent manner compared with the blank control group. As shown in Figure 12(b), the IC_50_ at 24 or 48 h is 31.99 ± 0.98 and 37.26 ± 0.97 *μ*g/mL, respectively.

### 3.9. Quercetin Induces G2/M Arrest in Human BRCA MDA-MB-231 Cells

In this study, flow cytometry was used to detect the effect of quercetin at different concentrations (0, 25, 30, 31.99, 35, and 40 *μ*g/mL) on the cell cycle of MDA-MB-231 cells for 24 h (Figure 13). Compared with untreated cells, the cells in the high concentration group of quercetin showed significant accumulation at the G2/M phase, indicating that quercetin blocked human BRCA MDA-MB-231 cells in the G2/M phase.

### 3.10. Quercetin Induces Apoptosis of Human BRCA MDA-MB-231 Cells and Activates p38MAPK Channel

In this study, flow cytometry was used to detect the effect of quercetin at different concentrations (0, 25, 31.99, 35, and 40 *μ*g/mL) on the apoptosis rate of MDA-MB-231 cells for 24 h (Figure 14). The total apoptosis rate of MDA-MB-231 cells in each quercetin group increased in a dose-dependent manner (*P* < 0.05), indicating that quercetin induced apoptosis in human BRCA MDA-MB-231 cells. The effect of quercetin on MDA-MB-231 apoptosis was further detected by western blotting. Caspase-3 and PARP are the core executive proteins in the apoptosis pathway, ERBB3 and MET are the screened core proteins, so the expression of these proteins was detected. As shown in Figure 15, quercetin increased the protein expression of cleaved caspase-3 and cleaved PARP in a dose-dependent manner (*P* < 0.05), indicating that quercetin may induce apoptosis of human MDA-MB-231 cells through caspase-3 and PARP. At the same time, ERBB3 and MET proteins decreased with the increase in quercetin concentration (*P* < 0.05). It is predicted that ERBB3 and MET could become biomarkers of quercetin, promoting MDA-MB-231 cell apoptosis. According to the results of KEGG pathway, the p38MAPK pathway played an important role in the action of *P. vulgaris* against BRCA. Based on the abovementioned reasons, this study speculated that quercetin induced apoptosis in human BRCA MDA-MB-231 cells may be related to the p38 channel, so the expression of p38 protein was detected. Quercetin increased the expression of p38 in a dose-dependent manner (*P* < 0.05), suggesting that the p38MAPK pathway may be involved in the process of apoptosis.

## 4. Discussion

In recent years, the incidence of BRCA has increased worldwide. Approximately 30% of the cases are metastatic BRCA [24]. Early stages of BRCA often go undetected, leading to the progression of the disease. Recent studies have shown that flavonoids and sterols are the main antitumor active components of *P. vulgaris* [25, 26]. Kaempferol (PL2) is a polyphenolic antioxidant that inhibits proliferation and induces apoptosis of cancer cells. It has been found that the mechanism of its induced apoptosis is related to the phosphatidylinositol 3-kinase/protein kinase B (PI3k/FAK) signaling pathway [27], which can significantly inhibit the proliferation of BRCA SK-BR-3 cells, which may be related to the regulation of Notch1 and cleaved caspase-3 protein expression [28]. Soybean sterol (PL4) is widely distributed in various plants. It has been found that soybean sterol, as a representative of terpenoids from Ilex latifolia, can effectively inhibit the proliferation of MDA-MB-231 cells and promote the apoptosis of cells in MDA-MB-231 [29]. Delphinidin (PL5), as an important component of the development of BRCA, has been well known by many scholars. Studies have shown that cyclin D1, c-myc, and MMP-7 are overexpressed in BRCA [30]. Cordycepin can significantly reduce *β*-catenin and p-GSK-3*β* in BRCA MDA-MB-231 cells. The protein expression level of Wnt can significantly reduce Wnt/*β* expression of target genes c-myc, cyclin D1, and MMP-7 downstream of the catenin signaling pathway. Delphinidin can also reduce the expression level of MMP-7 in breast tumor tissues [31]. Meanwhile, cordycepin can induce apoptosis of HER-2 positive BRCA MDA-MB-453 and induce autophagy by inhibiting the AKT/mTOR pathway [32]. It can also induce G2/M cycle arrest and apoptosis of MDA-MB-453 and BT-474 cells by blocking the NFkB signaling pathway, thereby having an antiproliferative effect [33]. Luteolin (PL6), originally called 3′,4′,5,7-tetrahydroxyflavone, contains c6-c3-c6, benzene ring, oxygenated carbon ring, and a C2-C3 carbon double bond, which is an important structure for luteolin to play its biological role [34, 35].

Studies have shown that luteolin inhibits the growth and proliferation of colorectal cancer cells, BRCA cells, prostate cancer cells, gastric cancer cells, and hepatoma cells, as well as affects the activation of multiple signaling pathways associated with growth and proliferation [36–38]. It can induce the growth inhibition of BRCA cells and reduce the methylation level of the OPCML gene. Because of its natural origin and low toxicity, it has been used as a potential safe tumor adjuvant drug [39]. Morin (PL10) can significantly reduce inflammation-mediated apoptosis induced by dihydroxymethylbutyric acid (DMBA). Morin can also effectively inhibit the downregulation of Bax and the upregulation of Bcl-2. In addition, Morin can downregulate proinflammatory markers such as COX-2, NFkB, TNF-*α*, IL-2, and IL-1*β*. Some experiments also confirmed that Morin mediated mitochondrial apoptosis is related to the release of cytochrome C and the apoptosis signaling pathway. Therefore, these results further suggest that Morin may induce apoptosis of cancer cells and further prevent BRCA under the condition of DMBA induction, which suggests that Morin may be clinically used as a marker of BRCA prevention [40]. In this study, 11 active components of *P. vulgaris* against BRCA were screened by TCMSP and OB and DL parameters. Flavonoids and sterols were the key active components. This study also found that quercetin played an anti-BRCA role by acting on multiple targets. For the abovementioned reasons, quercetin was selected for subsequent cell experiments to study its potential mechanism. In conclusion, quercetin plays a role in antagonizing BRCA through a variety of active ingredients, reflecting the synergistic effect of multiple components of Chinese medicine.

In this study, 179 common targets of *P. vulgaris* and BRCA were collected. Among them, SCN5A, MAP2, and TOP2A were the core predictive targets. In humans, voltage-gated sodium channels (VGSC) have nine subtypes, namely Nav1.1–Nav1.9, with different functional characteristics. Nav1.5 belongs to TTX-R VGSC and SCN5A is the genotype encoding Nav1.5. At present, studies have reported that the functional expression of SCN5A is found in many malignant tumor cells, and its increased expression and activity are closely related to the malignant biological characteristics of some tumors, which may be involved in the occurrence and development of tumors [41]. An abnormal expression of SCN5A was detected in BRCA MDA-MB-231 cells and BRCA tissues with lymph node metastasis. SCN5A may be an early tumor marker and prognostic factor in BRCA. Fraser et al. [42] showed that the expression of SCN5A was 1800 times higher in the metastatic cell line MDA-MB-231 than in that of the highly metastatic BRCA MDA-MB-231 cells, which confirmed that there was a significant correlation between the expression of SCN5A and the occurrence and development of BRCA. MAP2 includes four subtypes: high molecular weight MAP2A and MAP2B, and low molecular weight MAP2C and MAP2D. Some studies have found that paclitaxel is an antimitotic anticancer agent that is effective for solid tumors. Its antitumor activity comes from the inhibition of microtubule depolymerization and the promotion of microtubule assembly. In terms of mechanism research, it was found that paclitaxel can promote the increase of affinity between MAP2 and tubulins, affect the depolymerization and assembly of microtubules, and exert its antitumor activity [43]. Studies have shown that MAP2 also expresses corresponding mRNAs and related peptides in pancreatic ductal adenocarcinoma. Microtubules are one of the targets of docetaxel. *In vivo* hydrolysis of MAP2 protein can increase the antitumor effect of docetaxel in pancreatic ductal adenocarcinoma [44]. DNA topoisomerase (TOP2A) has an important relationship with the occurrence, development, invasion, treatment, and prognosis of malignant tumors. As a DNA topoisomerase, it is essentially a protein and is closely related to tumor chemotherapeutic drug targets [45]. TOP2A is mainly distributed in the nucleus and participates in the cell cycle pathway, which is closely related to cell proliferation and apoptosis. The expression of TOP2A during cell division is specific. It begins to increase in the S phase of mitosis, reaches its maximum in the G2/M phase, and decreases after division. BRCA is often associated with a high expression of the epidermal growth factor receptor (HER2/neu), while the TOP2A encoding gene is located at HER217/neu, and TOP2A expression is correlated with HER2/neu gene expression. Some scholars have found that the expression of HER2/neu and TOP2A is related to anthracycline chemotherapy. It is proven that the expression of these two genes can provide the basis for the selection of chemotherapeutic drugs for BRCA [46]. In addition, researchers have found a correlation between the expression of the TOP2A gene and the clinicopathological features of BRCA. The results provide the basis for anthracycline chemotherapy in the treatment of BRCA [47, 48]. Therefore, the expression of TOP2A can predict the effect of chemotherapy on BRCA. In summary, these targets are the important targets of *P. vulgaris* against BRCA, which reflect the synergistic effect of multiple targets.

In this study, KEGG pathway analysis showed that *P. vulgaris* exerts anti-BRCA effects through multiple signals, including the PI3K-Akt signaling pathway, the MAPK signaling pathway, and the AGE-RAGE signaling pathway. The PI3K/Akt signaling pathway promotes BRCA formation through a variety of cell processes, including promoting cell growth, proliferation, viability, transforming glycolysis metabolism, increasing cell migration, and reducing cell apoptosis [49]. PI3K signaling activates Akt kinase, activated Akt can be found in BRCA collection samples of 20% to 55%, and is related to the recurrence of ER-positive BRCA [50, 51]. The PI3K pathway mutation is the most common gene mutation in HR-positive BRCA and is found in over 70% of BRCA patients [52]. In recent studies on The Cancer Genome Atlas, 36% of BRCA had PIK3CA mutation [53], but PIK3CA mutation as a marker of prognosis of BRCA still has some controversies, which may be related to a small sample size [54]. Because PIK3CA encodes PI3K and catalyzes the subunit P110, it is meaningful to use inhibitors for specific PI3K subtypes in the development of PI3K inhibitors for the treatment of BRCA. In recent years, a large number of studies have shown that the level of advanced glycosylation end products (AGEs) in diabetics is significantly higher than that in the general population, and by inhibiting glycosylation, the progression of diabetic nephropathy can be effectively curbed. AGEs are a combination of receptors for AGEs (RAGE) and a series of lesions. A large number of studies have shown that the AGE-RAGE signaling pathway is a very important link in the formation and progression of diabetic nephropathy. However, its downstream mechanism is very complex and has still not been fully clarified such as NF-KB, VGEF, and TGF-*β*1. The relationship between the MCP-1 gene and other genes needs to be confirmed by further research.

ERBB3 plays an important role in the development of normal breast tissue. The expression level of ERBB3 is very low in normal breast tissue in the embryonic stage. Through the process of postnatal maturation, the expression of ERBB3 increases. In the second and third trimesters of pregnancy, it can be observed that the phosphorylation level increases after ERBB3 is activated, and the expression of ERBB3 also increases in the mammary duct epithelium and stroma of pregnant rats. In functionally differentiated or nontransformed breast epithelial cells, the expression and activation of ERBB3 are downregulated [55]. ERBB3 was not activated in the established normal immortalized breast cell line. About 35% of BRCA cell lines express a high level of ERBB3 compared to the nontransformed mammary cell line [56]. In human BRCA tissue samples, the expression of ERBB3 mRNA was increased by 100 times compared with normal breast tissue in 46% of the samples by RT-PCR [57]. 2D-PAGE protein analysis of four normal breast samples and four BRCA samples from humans revealed that ERBB3 was detected only in malignant tissues. Cancer tissues had higher ERBB3 expression than normal tissues in 50%–70% of BRCA cases. In 18%–29% of cases, the high expression of ERBB3 was positively correlated with metastasis, tumor size, in situ recurrence, tumor grade, and tumor recurrence. The ERBB2-ERBB3 heterodimer is considered to be the most interactive dimer form in the ERBB family. In the mouse model experiment, ERBB3 expression was also increased in ERBB2-induced tumors. The same situation was also observed in human BRCA. The amplification of ERBB2 was accompanied by an increase in ERBB3 expression [58].

Further studies have found the importance of ERBB3 in ERBB2 transformed cells. When ERBB3 expression is inhibited, ERBB2 cannot effectively transform cells [59]. Although EGFR and ERBB2 have no sites directly connected to PI3K, ERBB3 has seven. When it forms dimers with EGFR or ERBB2, it can phosphorylate and activate the PI3K signal transduction pathway [60]. Compared with other receptor combinations, ERBB2-ERBB3 coexpression increases the level of THE vascular endothelial growth factor in the cells [61]. Notably, in the invasive tumors caused by ERBB2 and ERBB3, THE insulin-like growth factor 2 (IGF2) and insulin-like growth factor binding protein 5 (IGFBP-5) are highly expressed, and these growth factors are very important for tumor growth [62]. Cellular mesenchymal to the epithelial transition factor (MET), also known as c-Met, is the product encoding the proto-oncogene MET. Its associated signaling pathway is closely related to the prognosis and drug resistance of BRCA and is an important potential therapeutic target for triple-negative BRCA [63–68]. Numerous studies have shown that the positive rate of c-Met in BRCA tissues is significantly higher than that in BRCA tissues. Its positive expression is closely related to the degree of differentiation, infiltration, lymph node metastasis, and clinical stages. It also indicates that the progression of BRCA is related to the activation of the c-Met proto-oncogene [69]. A study on the correlation between c-Met expression and BRCA in foreign countries has also confirmed that activated c-Met can induce mouse BRCA. This kind of BRCA is similar to human basal-like BRCA. It is characterized by PR (−), HER-2 (−), and CK5 (+). The high expression of c-Met protein indicates a poor prognosis and a significant negative correlation with the survival rate of BRCA [70]. Therefore, c-Met can be used as an important prognostic marker for patients with basal-like BRCA and has a significant prognostic value [71].

The MAPK signaling pathway plays an irreplaceable role in the proliferation, growth, and differentiation of breast tumor cells. It is a serine/threonine protein kinase widely found in eukaryotic cells. It can phosphorylate some target proteins and activate a series of cascade reactions to produce some biological effects in cells. The MAPK signaling pathway can transduce extracellular stimulation signals into cells and nuclei through a three-level kinase cascade: extracellular signal ⟶ MAPK kinase ⟶ MAPK kinase ⟶ MAPK. This pathway is involved in the processes of cell proliferation, growth, and apoptosis, and plays an important role in the occurrence and development of a variety of tumors. Filardo and Gper have shown that in NER-negative SKBR3 BRCA cells, estrogen can accelerate the phosphorylation of ERK1/2 and promote the proliferation of cancer cells [72]. Moreover, estrogen can activate ERK1/2 in MDA-MB-231 cells in a short time. Activation of the MAPK signaling pathway may affect the expression level and invasiveness of ER in BRCA cells. The expression of phosphorylated MAPK in normal breast tissues is significantly lower than that in BRCA tissues. Estrogen can not only promote the proliferation of BRCA cells through ER, but also activate the MAPK signaling pathway to induce tumor cell proliferation. In addition, the activation and expression of the p38-MAPK signaling pathway in lymph node-infiltrating breast tumors are more common than those in lymph node-negative breast tumors. In ER-negative BRCA MDAMB-468 and MDA-MB-231 cells in TGF-2*α* stimulated by serum, the level of ERK/MAPK phosphorylation and activity duration in cells were higher than those in ER-positive BRCA cell MCF-7, indicating that ERK/MAPK activation can promote the invasive growth of tumor cells. Song et al. found that in MCF-7, estrogen can produce rapid induction by binding with mer, activate SHC to form a SHC-GRB2-sos complex, activate the MAPK signal pathway, and finally affect the normal cycle of cell growth and abnormal proliferation of breast cells [73]. At the same time, researchers in our country have found that some Chinese medicine therapies may inhibit BRCA by regulating the ERK/MAPK signaling pathway. After the action of nitidine chloride on human BRCA cells, it was found that the drug could significantly reduce the expression levels of p-ERK1/2, p-JNK, and p-p38, indicating that nitidine chloride could inhibit the activity of the MAPK signaling pathway and inhibit the metastasis of breast tumors. Wang and Hu used the combination of Poria cocos triterpene and total iridoid of sepulchrysoides to observe the effect of the invasion ability of breast cancer cells [74]. Jingjing et al., in the study of Poria cocos triterpenes and ajiro total iridoid two drugs on the invasive ability of BRCA cells, found that high metastatic BRCA cells MDA-MB-231 and SK-BR-3 ERK1/2, JNK, and the p38 phosphorylation level were lower than before the combination. It is presumed that the combination of two drugs may inhibit the MAPK related signal transduction. It can hinder the invasion and metastasis of cancer cells. Other studies have confirmed that the Shugan Yishen recipe can reverse the expression of the HER-2 gene in BRCA cells and inhibit the two pathways of ERK/MAPK and p38/MAPK, thereby reversing the drug resistance of tumor cells [75, 76].

The study also has some limitations. First, the public database is updated in real time, so the results of this study only reveal to a certain extent the mechanism of *P. vulgaris* against BRCA. Second, this study was only carried out *in vitro* and only used human BRCA MDA-MB-231 cells. In future, further multidimensional validation is needed. It is very meaningful to study the effect of *P. vulgaris* on the role of anti-BRCA through various signaling pathways. For future research, the MAPK signaling pathway can be selected, and other signaling pathways, such as the PI3K-AKT signaling pathway, can be further studied. In addition, although quercetin is the main active component of *P. vulgaris*, it still cannot fully represent *P. vulgaris*, which still needs further experimental verification in the future. In conclusion, the mechanism of *P. vulgaris* against BRCA should be further studied *in vivo* and *in vitro*.

In this study, the potential mechanism of *P. vulgaris* against BRCA was preliminarily investigated by using network pharmacology, molecular docking, and *in vitro* experiments. The results showed that *P. vulgaris* played an important role in anti-BRCA through multicomponent, multitarget, and multisignal channels. Quercetin played an important role in this process. In addition, quercetin can effectively inhibit the proliferation of human BRCA cell MDA-MB-231 by regulating cell apoptosis and the cell cycle, which may be related to the MAPK signaling pathway. This study provides new inspiration for future experimental and clinical treatment of BRCA.

## Figures and Tables

**Figure 1:** Overall flow chart of the study.

**Figure 2:** Venn map of the common target of *Prunella vulgaris* and BRCA.

**Figure 3:** “Single-substance drug-disease-component-target” network of *Prunella vulgaris* L.

**Figure 4:** Interaction network of *Prunella vulgaris* against potential targets of BRCA.

**Figure 5:** Number of adjacent targets in the top 35.

**Figure 6:** Top 10 GO enrichment analysis histograms and scatter plots of the common targets of *Prunella vulgaris* and BRCA.

**Figure 7:** Top 10 KEGG pathway analysis histograms and scatter plots of the common targets of *Prunella vulgaris* and BRCA.

**Figure 8:** “Single-substance drug-component-disease-target-pathway” network of *Prunella vulgaris*.

**Figure 9:** Interaction between quercetin and receptor molecules.

**Figure 10:** Illustration of the MAPK signaling pathway.

**Figure 11:** Expression levels of ERBB3/MET in different tissues in the human protein database.

**Figure 12:** Effect of the concentration and action duration of quercetin on the viability of MDA-MB-231 cells (MTT). Error bars represent mean ± SD. ^*∗*^*P* < 0.05, ^*∗∗*^*P* < 0.01, vs. control.

**Figure 13:** Effect of quercetin on the MDA-MB-231 cell cycle. Error bars represent mean ± SD. ^*∗*^*P* < 0.05, ^*∗∗*^*P* < 0.01, vs. control.

**Figure 14:** Effect of quercetin treatment of MDA-MB-231 cells for 24 h on the apoptosis rate. Error bars represent mean ± SD. ^*∗*^*P* < 0.05, ^*∗∗*^*P* < 0.01, vs. control.

**Figure 15:** Effect of quercetin on cleaved caspase-3, cleaved PARP, ERBB3, MET, and p38 protein levels in MDA-MB-231 cells after 24 h of treatment. Error bars represent mean ± SD. ^*∗*^*P* < 0.05, ^*∗∗*^*P* < 0.01, vs. control.

**Table 1:** Active components of *Prunella vulgaris*.

Number	Molecule ID	Name	Oral bioavailability (OB)%	Drug-likeness (DL)
PL1	MOL000358	Beta-sitosterol	36.91391	0.75123
PL2	MOL000422	Kaempferol	41.88225	0.24066
PL3	MOL004355	Spinasterol	42.97937	0.75534
PL4	MOL000449	Stigmasterol	43.82985	0.75665
PL5	MOL004798	Delphinidin	40.63498	0.27763
PL6	MOL000006	Luteolin	36.16263	0.24552
PL7	MOL006767	Vulgaxanthin-I	56.13969	0.25836
PL8	MOL006772	Poriferasterol monoglucoside_qt	43.82985	0.75769
PL9	MOL006774	Stigmast-7-enol	37.42312	0.75133
PL10	MOL000737	Morin	46.22959	0.27457
PL11	MOL000098	Quercetin	46.43335	0.27525

**Table 2:** Binding energy between quercetin and the top 10 targets in the PPI network.

Receptor	Pub ID	Binding energy/kcal·mol^−1^	Basic binding energy/kcal·mol^−1^
ERBB3	3kex	−9.1	−7.56
INSR	2hr7	−7.3	−6.97
MET	2rfs	−8.2	−7.84
NCOA1	2c52	−5.8	−5.51
NCOA2	5egv	−4.8	−4.42
COL3A1	6fzw	−6.6	−6.31
TOP2A	4r1f	−8.4	−7.12
DUOX2	AF	−8	−7.24
MAP2	AF	−6	−5.62
SCN5A	6lqa	−7.8	−7.31

## Data Availability

The datasets used and/or analyzed during the study are available from the corresponding author upon request.
